# Discussion on Repolarization Reserve between Patients with Coronary Heart Disease and Normal Controls

**DOI:** 10.1155/2022/7944969

**Published:** 2022-08-18

**Authors:** Rubing Kang, Yitong Li, Chunmei Gao, Jianhui Li, Cheng Zhang, Junli Wang

**Affiliations:** ^1^Department of Cardiology, Heji Hospital Affiliated to Changzhi Medical College, Changzhi, 046011 Shanxi, China; ^2^Guizhou Medical University, Guiyang, 550025 Guizhou, China; ^3^Department of ECG Diagnosis, Second Hospital of Shanxi Medical University, Taiyuan, 030001 Shanxi, China; ^4^Department of Cardiology, Binhai Hospital of Peking University (Tianjin Fifth Central Hospital), Tianjin 300450, China

## Abstract

**Objective:**

To investigate the repolarization reserve of normal controls (NCs) and patients with coronary heart disease (CHD).

**Methods:**

From January 1st, 2010 to December 31st, 2018, 200 age- and gender-matched inpatients in the Second Hospital of Shanxi Medical University and Heji Hospital Affiliated to Changzhi Medical College were selected for treadmill exercise test (TET), including 67 patients in the myocardial ischemia group, 66 patients in the suspected myocardial ischemia group, and 67 patients in the normal control group. Coronary angiography (CAG) was performed on 49 of 133 patients in the myocardial ischemia group and the suspected myocardial ischemia group, and 9 positives and 40 negatives were identified. The heart rate (HR) and QT interval of TET examiners before exercise, during exercise (90 beats/min, 120 beats/min, maximum HR), and in the recovery period (1 minute and 3 minutes after exercise) were reviewed, and QTc values were calculated after being corrected by BaZett's.

**Results:**

The mean QTc values in NCs were all below 452 ms, before exercise, during exercise (90 beats/min, 120 beats/min and maximum HR), and during the recovery period (1 minute and 3 minutes after exercise). The comparison results of the RR interval between the two groups revealed *P* > 0.05, indicating no statistical significance. Significant differences were present when comparing the QT intervals when the HRs were 90 beats/minute and 120 beats/minute during exercise (*P* < 0.05). And comparing the QTc values, it was found that the QTc values during different exercise periods were statistically different between groups (*P* < 0.05).

**Conclusions:**

NCs have good repolarization reserve. CAG can confirm true myocardial ischemia patients (i.e., patients with CHD) among myocardial ischemia and suspected myocardial ischemia patients screened by TET. Patients with positive CAG have poor repolarization reserve as QT interval represents ventricular repolarization adaptability.

## 1. Introduction

It is well known that human ventricular repolarization (interval) is inversely proportional to heart rate [1, 2]. When the heart rate is fast, the ventricular repolarization period is shortened while significantly prolonged when the heart rate is slow [3, 4]. This kind of frequency adaptability of ventricular repolarization which is called ventricular repolarization reserve, also known as ventricular repolarization adaptability, is of great significance to the automatic regulation and effectiveness of ventricular contraction and relaxation under physiological conditions [5, 6]. In recent years, evidences have shown that the inward late sodium current in the plateau phase of cell membrane plays a key role in the frequency adaptation of ventricular repolarization [7–9]. Meanwhile, we also found that the late sodium current, as an important inward current in the plateau phase of action potential, is very sensitive to the stimulation frequency [10]. When the stimulation frequency is fast, the current is small; otherwise, it is the opposite [11].

A large number of studies have shown that myocardial ischemia from different causes, such as heart failure [12], myocardial infarction [13], cardiomyopathy [14], and myocarditis [15], can lead to the reduction of repolarization reserve capacity, which becomes acquired long QT syndrome [16]. The primary reason for this was that slow delayed rectifier potassium current (Iks) is an important repolarization reserve of human cardiomyocytes [17]. The decrease of outward current or the increase of inward current caused by myocardial ischemia, or both, can reduce the ventricular reserve function and prolong the interval [18]. Moreover, the formation of late sodium current and the change of early and late depolarization potential can synergistically lead to malignant arrhythmia and eventually cardiac death on the basis of the reduction of existing myocardial repolarization reserve [19].

The treadmill exercise test [20] in this study is a simple and relatively safe, noninvasive test for the diagnosis of myocardial ischemia, and it is a test to increase cardiac load through exercise. The functional state of the heart was determined by the principle that the body should increase coronary blood flow correspondingly when exercising, which can find myocardial ischemia caused by various reasons. The novelty and motivation of this study is to use such principle to make the patients stop when the maximum heart rate of the exercise test reaches the symptom limitation by means of passive exercise and compares the interphase changes and change rules of the patients in the recovery period before exercise and after exercise to determine whether the function of repolarization reserve is impaired. The research results are reported as follows.

## 2. Methods

### 2.1. Research Participants

From January 1st, 2010 to December 31st, 2018, 200 inpatients in the Second Hospital of Shanxi Medical University and Heji Hospital Affiliated to Changzhi Medical College were selected for treadmill exercise test (TET), including 67 patients in the myocardial ischemia group (positive group), 66 patients in the suspected myocardial ischemia group (suspected positive group), and 67 patients in the normal control group (negative group). Forty-nine of the 133 cases in the myocardial ischemia group and suspected myocardial ischemia group underwent coronary angiography (CAG), of which 9 cases were positive and 40 cases were negative. This study was approved by the Ethics Committee of Heji Hospital affiliated to Changzhi Medical College.

### 2.2. Data Collection

The heart rate (HR) and QT interval of TET examiners before exercise, during exercise (90 beats/min, 120 beats/min, maximum HR), and during the recovery period (1 minute and 3 minutes after exercise) were reviewed, and QTc values were calculated after BaZett's correction. CAG, the “golden standard” for diagnosing coronary heart disease (CHD), has been extensively used in clinical practice, by which positive and negative patients were further diagnosed in this study. The repolarization reserve function of positive and negative patients was judged by the comparison of RR interval, QT interval, and QTC values. In the following, the repolarization reserve of normal controls (NCs) and the difference between patients with positive CAG and those with negative CAG were studied by TET.

### 2.3. Instruments and Methods

#### 2.3.1. Treadmill Exercise Test

Q-stress Treadmill produced by Quinton, USA was used. Medication that may cause abnormal ST segment changes and elevated myocardial oxygen consumption was discontinued three days before the examination, and smoking and alcohol were prohibited after meals or 2 hours before meals. The Bruce's protocol was adopted, that is, the test was terminated at 85% of the expected maximum HR for age (220-age). Multidirectional and multiangle selective left and right CAG was performed by percutaneous puncture into the femoral artery of the lower extremities with the use of a C-arm machine. The left coronary artery was projected in at least four positions, with at least two positions of the coronary artery, and additional positions as necessary to fully reveal the segments of the coronary artery. Diagnostic criteria are as follows: CHD was confirmed if the CAG showed at least 1 lumen stenosis ≥50% in the left main artery, left anterior descending artery, left circumflex artery, and right coronary artery.

#### 2.3.2. Repolarization Reserve

The HR and QT intervals of TET examiners were measured before exercise, during exercise (90 beats/minute, 120 beats/minute and maximum HR), and in the recovery period (1 minute and 3 minutes after exercise), and their changes were compared. $\text{QTc}=\text{QT interval}/\sqrt{RR\text{ interval}}$ interval; the smaller the QTc value, the better the repolarization reserve.

#### 2.3.3. Measurement Methods

In all the three groups, consecutive RR intervals before exercise, during exercise (90 beats/min, 120 beats/min, maximum HR), and in the recovery period (1 minute and 3 minutes after exercise) were selected for manual measurement of RR and QT intervals. The lead with T wave amplitude at least greater than 2 mm and clear T wave end in the routine-lead was selected. For the same patient, the same lead was always measured. In some cases where the end of T wave was difficult to identify (biphasic T wave, T wave notch, T-U wave fusion, etc.), a tangent line was drawn from the steepest part of the descending branch of T wave crest, and the intersection of this tangent line and equipotential line was considered the end of T wave. In patients with bundle branch block, the QRS time difference before and after block was subtracted to adjust the QT interval.

### 2.4. Statistical Processing

Data analysis was performed by SPSS17.0. Categorical data were expressed by mean ± standard deviation (SD), while measurement data were expressed by *n* (%). The differences in the RR interval, QT interval, and QTc values among two groups were identified by the independent sample *t*-test; statistical comparisons of the groups were conducted using one-way ANOVA, with *P* < 0.05 as the significance level.

## 3. Results

### 3.1. RR Interval, QT Interval, and QTc Values in Normal Controls

In NCs, RR interval and QT interval were shortened with the increase of treadmill speed. However, as the postexercise recovery period increased, RR interval and QT interval were gradually prolonged. The mean QTc values were all below 452 ms (Table 1 and Figure 1).

### 3.2. Comparison of Age and Sex Composition between Groups

This study also compared the age and gender composition between NCs and patients with positive CAG for statistically analysis. The results showed *P* > 0.05, indicating no significant difference between groups (Table 2).

### 3.3. RR and QT Intervals and QTc Values of Patients with Normal Control and Negative and Positive CAG

The RR interval differences between the normal control group and negative CAG and positive CAG patients before exercise, when the HR was 90 beats/min during exercise, 120 beats/min during exercise or with maximum HR during exercise, all showed no statistical significance (*P* > 0.05). However, the RR intervals of the patients with negative CAG were significant lower that those in the normal control group (*P* < 0.05). One minute after exercise and at 3 minutes after exercise, the RR intervals of the normal control group and patients with negative and positive CAG suggested the absence of statistical significance (*P* > 0.05).

The comparison of preexercise QT intervals in the normal control and negative and positive CAG patients indicated statistical significance (*P* < 0.05). While the QT intervals in the normal control and negative and positive CAG patients with different HRs during exercise showed that the QT interval at the HR of 90 beats/minute and 120 beats/minute during exercise was statistically different between three groups (*P* < 0.05), the data showed no obvious difference in the QT interval between three groups at one minute after exercise (*P* > 0.05) and obvious difference in 3 minutes after exercise.

The differences of preexercise QTc values in the control, negative, and positive CAG patients indicated the presence of statistical significance (*P* < 0.05). It also showed that the QTc values were statistically different between patients with negative CAG and those with positive CAG during exercise (*P* < 0.05). The QTc values in patients at one minute after exercise showed obvious difference between groups (*P* < 0.05), while the data at 3 minutes after exercise presented no obvious difference between groups (*P* > 0.05), as shown in Tables 3 and 4 and Figure 2.

## 4. Discussion

The generation of myocardial action potential is the result of sequential activation and deactivation of inward sodium and calcium ion currents and various outward potassium currents on myocardial cell membrane [21]. Experimental studies in the 1980s [22–25] have reached an important conclusion, that is, when the outward current decreases and/or the inward current increases, early postdepolarization will occur, resulting in the prolongation of action potential duration. At the same time, it is recognized that window calcium current plays an important role [26]. In this case, the L-type calcium channels may reactivate and reverse repolarization during action potential platform [27]. Physiologically, potassium ion current constitutes the main ion current of repolarization and exits through different potassium ion channels on the cell membrane. It is the repolarization potential of these different potassium ion currents that constitutes the basic repolarization reserve [28]. Under normal circumstances, human ventricular repolarization period (QT interval) is directly proportional to RR interval and inversely proportional to HR, that is, the ventricular repolarization period is shortened when the HR is fast, and significantly prolonged when the HR is slow [29]. The findings of this study fully conform to this law. Patients with myocardial ischemia and suspected myocardial ischemia were screened by TET, and the true positives were further confirmed by CAG. Significant differences were found when retrospectively comparing the QTc values of patients with positive and negative CAG. Since QT interval represents ventricular repolarization adaptability, this result indicates that patients with positive CAG have poor repolarization reserve capacity. This is because the main current of action potential repolarization of ventricular myocytes is formed by potassium ions flowing out of different kinds of potassium channels. Phase-1 repolarization is participated by IKto (instantaneous outward potassium current); phase-2 and 3 repolarization involves IKR (rapidly delayed rectifier potassium current) and IKS (slow delayed rectifier potassium current), and; phase-3 and 4 repolarization consists of IK1 (inward rectifier potassium current)[30]. The main factor affecting potassium efflux is the functional state of potassium channels, which can determine the characteristics of cell action potential repolarization and reduce potassium efflux by inhibiting the function of potassium channels. There is remodeling of cardiac repolarization in myocardium of myocardial ischemia caused by various reasons, and repolarization originates from the remodeling of ion channels and ion currents in cardiomyocytes [31]. Moreover, the current remodeling of ion channels in ischemic cardiomyocytes is mainly due to the reduction and downregulation of Ito and Ik1 currents, especially the slow activation of Iks channels, which can cause the change of cardiac repolarization into acquired long QT syndrome and reduce repolarization reserve [32].

In this study, we used the treadmill exercise test for the diagnosis of myocardial ischemia, and it is a test to increase cardiac load through exercise. However, when conducting exercise tests, the inadaptability to exercise or excessive load will produce undefined changes, which will affect the test results. Therefore, whether the test is carried out on the treadmill or on the circulatory power meter, it must always adapt to the clinical and biomechanical conditions of patients, so as to accurately explain the clinical variables.

## 5. Conclusion

The QT interval of patients with positive CAG does not decrease with the increase of ventricular rate, that is, the ventricular repolarization period is inversely proportional to the HR. When the HR increases, the ventricular repolarization period does not shorten correspondingly, but prolongs, indicating poor repolarization reserve capacity in patients with positive CAG.

## Figures and Tables

**Figure 1:** Change trends during RR and QT in the normal group.

**Figure 2:** Comparison of RR interval, QT interval, and QTc value between patients with the normal control and positive and negative coronary angiography ($\bar{x}\pm s$). (a) Initial heart rate before exercise. (b) 90 beats/minute during exercise. (c) 120 beats/minute during exercise. (d) Maximum heart rate during exercise. (e) During the recovery period 1 minute after exercise. (f) During the recovery period 3 minute after exercise. ^∗^*P* < 0.05, compared to the normal control group; ^#^*P* < 0.05, compared to the negative CAG group).

**Table 1:** RR interval and QT intervals as well as QTc values of normal controls during different exercise periods ($\bar{x}\pm s$).

Index	Value
Number	67
Age	52.22 ± 9.31
Before exercise	
RR interval	777.79 ± 118.74
QT interval	399.07 ± 31.44
QTc value	454.78 ± 27.16
90 beats/minute during exercise	
RR interval	663.79 ± 3.91
QT interval	371.90 ± 19.11
QTc value	456.39 ± 23.89
120 beats/minute during exercise	
RR interval	498.13 ± 5.53
QT interval	335.42 ± 16.25
QTc value	475.36 ± 22.97
Maximum heart rate during exercise	
RR interval	432.13 ± 46.63
QT interval	307.34 ± 22.49
QTc value	467.76 ± 28.01
During the recovery period (1 minute after exercise)	
RR interval	511.06 ± 70.03
QT interval	330.93 ± 28.25
QTc value	466.72 ± 22.92
During the recovery period (3 minute after exercise)	
RR interval	647.28 ± 121.96
QT interval	368.19 ± 31.27
QTc value	461.49 ± 28.14

**Table 2:** Comparison of age and sex composition between two groups ($\bar{x}\pm s$).

	Age	Gender (male/female)
Negative coronary angiography (*n* = 40)	55.18 ± 10.20	22/18
Positive coronary angiography (*n* = 9)	51.44 ± 14.22	5/4
*t*/*x*^2^	0.923	0.001
*P*	0.361	0.976

There was no significant difference between the two groups (*P* > 0.05).

**Table 3:** Comparison of RR interval, QT interval, and QTc value between patients with positive and negative coronary angiography ($\bar{x}\pm s$).

Index	Negative CAG (*n* = 40)	Positive CAG (*n* = 9)	*t*	*P*
Initial heart rate (before exercise)				
RR interval	751.38 ± 75.82	750.33 ± 109.20	0.035	0.973
QT interval	389.30 ± 25.05	419.22 ± 48.78	2.665	0.011
QTc value	451.25 ± 37.63	485.56 ± 31.67	2.535	0.014
90 beats/minute during exercise				
RR interval	663.43 ± 3.90	665.22 ± 4.06	1.235	0.223
QT interval	367.25 ± 13.23	387.78 ± 18.34	4.132	0.000
QTc value	450.93 ± 16.42	475.22 ± 23.39	3.699	0.001
120 beats/minute during exercise				
RR interval	499.85 ± 4.67	498.11 ± 4.94	0.999	0.323
QT interval	323.30 ± 11.27	342.56 ± 20.34	3.937	0.000
QTc value	457.43 ± 16.11	485.33 ± 27.78	4.061	0.000
Maximum heart rate during exercise				
RR interval	414.08 ± 31.85	419.56 ± 54.31	0.405	0.687
QT interval	291.60 ± 26.14	308.89 ± 24.47	1.812	0.076
QTc value	448.75 ± 20.53	476.67 ± 24.50	3.560	0.001
During the recovery period (1 minute after exercise)				
RR interval	514.03 ± 65.06	504.56 ± 85.01	0.373	0.711
QT interval	319.30 ± 23.44	331.11 ± 31.40	1.282	0.206
QTc value	446.75 ± 23.69	470.00 ± 25.98	2.615	0.012
During the recovery period (3 minute after exercise)				
RR interval	643.92 ± 116.71	643.00 ± 98.91	0.022	0.983
QT interval	351.75 ± 30.23	381.44 ± 41.30	2.485	0.017
QTc value	442.50 ± 28.80	474.44 ± 27.89	3.022	0.004

There were significant differences in QTc values among the three groups (*P* < 0.05).

**Table 4:** Comparison of RR interval, QT interval, and QTc value between patients with normal control, positive, and negative coronary angiography ($\bar{x}\pm s$).

Index	Normal control (*n* = 67)	Negative CAG (*n* = 40)	Positive CAG (*n* = 9)	*F*	*P*
Initial heart rate (before exercise)					
RR interval	777.79 ± 118.74	751.38 ± 75.82	750.33 ± 109.20	0.906	0.407
QT interval	399.07 ± 31.44	389.30 ± 25.05	419.22 ± 48.78^b^	3.686	0.028
QTc value	454.78 ± 27.16	451.25 ± 37.63	485.56 ± 31.67^ab^	4.475	0.014
90 beats/minute during exercise					
RR interval	663.79 ± 3.91	663.43 ± 3.90	665.22 ± 4.06	0.768	0.466
QT interval	371.90 ± 19.11	367.25 ± 13.23	387.78 ± 18.34^ab^	5.241	0.007
QTc value	456.39 ± 23.89	450.93 ± 16.42	475.22 ± 23.39^ab^	4.690	0.011
120 beats/minute during exercise					
RR interval	498.13 ± 5.53	499.85 ± 4.67	498.11 ± 4.94	1.434	0.243
QT interval	335.42 ± 16.25	323.30 ± 11.27^a^	342.56 ± 20.34^b^	10.580	0.000
QTc value	475.36 ± 22.97	457.43 ± 16.11^a^	485.33 ± 27.78^b^	11.450	0.000
Maximum heart rate during exercise					
RR interval	432.13 ± 46.63	414.08 ± 31.85^a^	419.56 ± 54.31	2.308	0.104
QT interval	307.34 ± 22.49	291.60 ± 26.14^a^	308.89 ± 24.47	5.809	0.004
QTc value	467.76 ± 28.01	448.75 ± 20.53^a^	476.67 ± 24.50^b^	8.651	0.000
During the recovery period (1 minute after exercise)					
RR interval	511.06 ± 70.03	514.03 ± 65.06	504.56 ± 85.01	0.073	0.930
QT interval	330.93 ± 28.25	319.30 ± 23.44^a^	331.11 ± 31.40	2.452	0.091
QTc value	466.72 ± 22.92	446.75 ± 23.69^a^	470.00 ± 25.98^b^	9.983	0.000
During the recovery period (3 minute after exercise)					
RR interval	647.28 ± 121.96	643.92 ± 116.71	643.00 ± 98.91	0.013	0.987
QT interval	368.19 ± 31.27	351.75 ± 30.23^a^	381.44 ± 41.30^b^	4.911	0.009
QTc value	461.49 ± 28.14	442.50 ± 28.80^a^	474.44 ± 27.89^b^	7.694	0.000

Note: ^a^comparison with the normal control, *P* < 0.05; ^b^comparison with negative CAG, *P* < 0.05.

## Data Availability

The labeled datasets used to support the findings of this study are available from the corresponding author upon request.
